This article has been retracted.

# Identification of Novel SCN5A Single Nucleotide Variants in Brugada Syndrome: A Territory-Wide Study From Hong Kong

**DOI:** 10.3389/fphys.2020.574590

**Published:** 2020-09-18

**Authors:** Gary Tse, Sharen Lee, Tong Liu, Ho Chuen Yuen, Ian Chi Kei Wong, Chloe Mak, Ngai Shing Mok, Wing Tak Wong

**Affiliations:** ^1^Xiamen Cardiovascular Hospital, Xiamen University, Xiamen, China; ^2^Tianjin Key Laboratory of Ionic-Molecular Function of Cardiovascular Disease, Department of Cardiology, Tianjin Institute of Cardiology, Second Hospital of Tianjin Medical University, Tianjin, China; ^3^Laboratory of Cardiovascular Physiology, Li Ka Shing Institute of Health Sciences, Faculty of Medicine, The Chinese University of Hong Kong, Shatin, China; ^4^Department of Medicine and Geriatrics, Princess Margaret Hospital, Kowloon, China; ^5^Centre for Safe Medication Practice and Research, Department of Pharmacology and Pharmacy, Li Ka Shing Faculty of Medicine, The University of Hong Kong, Pokfulam, China; ^6^School of Pharmacy, University College London, London, United Kingdom; ^7^Department of Pathology, Hong Kong Children’s Hospital, Kowloon, China; ^8^State Key Laboratory of Agrobiotechnology (CUHK), School of Life Sciences, The Chinese University of Hong Kong, Shatin, China

**Keywords:** Brugada syndrome, SCN5A, ventricular arrhythmias, risk stratification, Sudden cardiac death

## Abstract

**Background:**

The aim of this study is to report on the genetic composition of Brugada syndrome (BrS) patients undergoing genetic testing in Hong Kong.

**Methods:**

Patients with suspected BrS who presented to the Hospital Authority of Hong Kong between 1997 and 2019, and underwent genetic testing, were analyzed retrospectively.

**Results:**

A total of 65 subjects were included (*n* = 65, 88% male, median presenting age 42 [30–54] years old, 58% type 1 pattern). Twenty-two subjects (34%) showed abnormal genetic test results, identifying the following six novel, pathogenic or likely pathogenic mutations in SCN5A: c.674G > A, c.2024-11T > A, c.2042A > C, c.4279G > T, c.5689C > T, c.429del. Twenty subjects (31%) in the cohort suffered from spontaneous ventricular tachycardia/ventricular fibrillation (VT/VF) and 18 (28%) had incident VT/VF over a median follow-up of 83 [Q1–Q3: 52–112] months. Univariate Cox regression demonstrated that syncope (hazard ratio [HR]: 4.27 [0.95–19.30]; *P* = 0.059), prior VT/VF (HR: 21.34 [5.74–79.31; *P* < 0.0001) and T-wave axis (HR: 0.970 [0.944–0.998]; *P* = 0.036) achieved *P* < 0.10 for predicting incident VT/VF. After multivariate adjustment, only prior VT/VF remained a significant predictor (HR: 12.39 [2.97–51.67], *P* = 0.001).

**Conclusion:**

This study identified novel mutations in SCN5A in a Chinese cohort of BrS patients.

## Introduction

Brugada syndrome (BrS) is an ion channelopathy with significant genetic heterogeneity. The most common mutations are loss-of-function variants in SCN5A, the gene responsible for the α-subunit of the Na^+^ channel. Since 2001, more than 80 mutations in the SCN5A gene have been associated with BrS (Antzelevitch et al., 2005). Mutations in other genes encoding for K^+^, Ca^2+^ and hyperpolarization-activated cyclic nucleotide-gated (HCN) channels have also been described. This condition was believed to be a Mendelian disease with an autosomal dominant inheritance pattern and incomplete penetrance (Sicouri et al., 2012). However, recent evidence suggests that this may not be true (Gourraud et al., 2016). A study investigated co-segregation of SCN5A mutations amongst large genotyped families, demonstrating that some affected family members did not carry the familial mutation (Probst et al., 2009). Therefore, mutations in other genes may be responsible for BrS (Marian, 2009; Roden, 2010). Another possibility is incomplete penetrance despite the presence of the mutated gene or variable expressivity (Giudicessi and Ackerman, 2013). Whilst the genetic epidemiology of BrS has been extensively studied in Western populations (Meregalli et al., 2009; Hu et al., 2014; Baruteau et al., 2018; Robyns et al., 2018), data from Asian countries are less complete.

A large multicenter registry from Japan examined the genotype-phenotype correlation of SCN5A mutations in BrS, demonstrating that those with SCN5A mutations showed greater conduction abnormalities and arrhythmic risks (Yamagata et al., 2017). A study from a tertiary hospital in Thailand investigated the genetic makeup of 40 BrS patients with implantable cardioverter-defibrillator (ICD) implants, reporting that the SCN5A-R1193Q variant is associated with cardiac conduction disturbances (Makarawate et al., 2017). In a Korean study, 21 BrS patients or their family members underwent genetic testing, demonstrating SCN5A mutations in four patients (Shin et al., 2004). In Chinese cohorts, the data remain limited with few studies from Taiwan (Juang et al., 2003), Hong Kong (Mok et al., 2004; Mak et al., 2018), mainland China (Zhang et al., 2016), and Singapore (Tan et al., 2011). These were reported as case series or included only a subset of patients in a sudden death cohort. In this territory-wide study from Hong Kong, we analyzed the genetic makeup of BrS patients, who underwent genetic testing over a 21-year period.

## Methods

### Study Population

This retrospective study was approved by The Joint Chinese University of Hong Kong–New Territories East Cluster Clinical Research Ethics Committee (Reference number: 2019.338). This study included consecutive patients suspected of BrS undergoing genetic testing between 1997 and 2019 identified from a territory-wide search of the electronic health records managed by the Hospital Authority of Hong Kong. The diagnosis of BrS was confirmed by review of patient case notes and documented ECGs by SL and GT using the 2017 diagnostic criteria proposed by the Expert Consensus Statement (Antzelevitch et al., 2016). The joint guidelines from Heart Rhythm, European and Asian Society guidelines were adopted for drug challenge test due to the use of older guidelines in past practice. Diagnosis was confirmed by an expert clinical electrophysiologist (NM) with more than 20 years of cardiac electrophysiology experience. Type 1 (coved pattern) is defined as ascending and high take-off of ≥2 mm at the end of QRS duration, followed by coved or rectilinear down-sloping ST-segment, and negative symmetric T-wave in ≥1 right precordial lead, V1 and V2. Type 2 (saddle-back pattern) is defined as high take-off r′ of ≥2 mm, followed by convex ST-elevation remaining at ≥0.5 mm relative to isoelectric line, and positive T-wave in V2 (T_peak_ > ST_minimum_) or T-wave of variable morphology in V1.

Clinical data was extracted from the electronic health records. The following baseline clinical data were collected: (1) sex; (2) age of initial Brugada pattern presentation; (3) follow-up period; (4) type of Brugada pattern and presence of fever at initial presentation; (5) family history of BrS and ventricular tachycardia (VT), ventricular fibrillation (VF) or sudden cardiac death (SCD); (5) manifestation of syncope and if present, the number of episodes; (6) manifestation of VT/VF and if present, the number of episodes; (7) performance of sodium channel blocker challenge test, electrophysiological study (EPS), BrS-related genetic screening, and their respective results and (8) implantation of ICD. Incident VT/VF events were those that occurred after initial presentation to the hospital. Spontaneous VT/VF included events that occurred both before and after presentation.

### ECG Measurements

Automated measurements from baseline ECGs were extracted, including (1) heart rate; (2) P wave duration; (3) PR interval; (4) QRS duration; (5) QT and QTc interval; (6) P wave, QRS and T wave axis; (7) S-wave amplitude in lead V1 and R-wave amplitude in lead V5.

### Genetic Testing

Genomic DNA was extracted using a QIAamp Blood Kit (Qiagen, Hilden, Germany). The coding exons and the flanking introns (10 bp) of each gene were amplified by polymerase chain reaction (primer sequences and protocol available upon request). Sanger sequencing was performed for SCN5A gene. The pathogenicity of novel missense variants was analyzed by Alamut Visual (Interactive Biosoftware, Rouen, France) with Polymorphism Phenotyping v2 (PolyPhen-2), Sorting Intolerant from Tolerant (SIFT), MutationTaster, and Assessing Pathogenicity Probability in Arrhythmia by Integrating Statistical Evidence (APPRAISE)^1^ and that of novel splicing variants by Splice Site Finder-like, MaxEntScan, NNSPLIC, GeneSplicer, and Human Splicing Finder, wherever appropriate. Splicing variants were considered to be damaging if there was a >10% lower score when compared with the wild-type prediction. Allele frequencies among populations were referred to the Exome Aggregation Consortium (ExAC)^2^. Interpretation of genetic findings was made by an expert pathologist with a specialist interest in cardiovascular genetics (CM).

### Statistical Analysis and Risk Prediction

All statistical analysis was performed using Stata MP (Version 13.0). Categorical variables were expressed as total number (percentages). Continuous variables were expressed as mean ± standard deviation. Significant differences between groups were determined using the Fisher’s Exact test and the Wilcoxon rank sum test for categorical and continuous variables, respectively. *P*-value < 0.05 was considered statistically significant.

The primary outcome of this study was incident VT/VF. Follow-up duration was defined as the time difference (in months) between the initial date of Brugada pattern presentation and the first occurrence of VT/VF post-diagnosis. Univariate Cox regression was used to identify significant predictors of the primary outcome. Hazard ratios and their 95% confidence intervals (CIs) with the corresponding *P*-values are reported. Variables with *P* < 0.10 were included in the multivariate model. Kaplan-Meier survival curves were constructed for the significant variable(s) in multivariate Cox regression and significant differences were determined by the log-rank test.

## Results

### Baseline Characteristics and Genetic Findings

In this study, patients who were diagnosed with BrS (*n* = 545), and subsequently underwent genetic testing (*n* = 56; 88% male, median presenting age 42 [30–54] years old, 58% with a type 1 Brugada pattern) were included.

### Follow-Up and Predictors of Spontaneous VT/VF Outcomes Post-diagnosis

Over a median follow-up of 83 [Q1–Q3: 52–112] months, 18 (28%) patients developed incident VT/VF. There was no significant difference in VT/VF occurrence between genetic positive and negative groups. Univariate Cox regression was used to identify significant predictors. Syncope (hazard ratio [HR]: 4.27 [0.95–19.30]; *P* = 0.059), prior VT/VF (HR: 21.34 [5.74–79.31; *P* < 0.0001) and T-wave axis (HR: 0.970 [0.944–0.998]; *P* = 0.036) achieved *P* < 0.10. After multivariate adjustment, only prior VT/VF remained a significant predictor (HR: 12.39 [2.97–51.67], *P* = 0.001). A Kaplan-Meier curve demonstrating freedom from spontaneous VT/VF during follow-up stratified by prior VT/VF status is shown in Figure 1. Those with prior VT/VF had a higher risk of incident VT/VF (*P* < 0.001, log-rank test).

**FIGURE 1:** Kaplan-Meier curve demonstrating freedom from spontaneous ventricular tachycardia/ventricular fibrillation (VT/VF) during follow-up for patients with (red line) and without (blue line) prior VT/VF. *P* < 0.001 by the log-rank test.

## Discussion

The main findings of this study are the identification of novel mutations in SCN5A and one novel mutation in CACNA1C in a Chinese cohort of BrS patients, and demonstration of abnormal T-wave axis as a predictor of incident VT/VF. Previously, altered T-wave axis was found to predict SCD in a middle-age adult population (Aro et al., 2012). The focus of this discussion are the novel mutations detected by genetic testing. Those that were previously described in other cohorts are detailed in the Supplementary Appendix.

The voltage-gated Na^+^ channels are made of large α subunits associated with other proteins, such as β subunits (SCN1B, SCN2B, and SCN3B). The SCN5A gene encodes for the α-subunit of the cardiac sodium channel. Loss-of-function mutations in SCN5A have been associated with BrS (Chen et al., 1998; Christien Li et al., 2016; Lee et al., 2020), sick sinus syndrome (SSS) (Benson et al., 2003), progressive cardiac conduction defect (PCCD, or Lenègre-Lev disease) (Tan et al., 2001) and overlap disorders between these conditions (Remme et al., 2008). An international compendium of putative BrS-associated genetic mutations in SCN5A was published in 2010 (Kapplinger et al., 2010). This study identifies six novel mutations in SCN5A in BrS, which have not been reported in cohorts outside of our geographical region.

The c.674G > A mutation, which was previously described in a dilated cardiomyopathy cohort (Shen et al., 2017), leads to a reduction in the peak sodium current (Li et al., 2018). This is expected to reduce conduction velocity of the propagating cardiac potentials, predisposing to the development of ventricular arrhythmias by reentry. However, our one patient harboring this mutation also carried the c.677C > T SNP. He had a family history of BrS. However, despite having a spontaneous type 1 Brugada pattern, he had a negative EPS with no complaints. This mutation has been identified as causative for long QT syndrome type 3 (Millat et al., 2006). Another variant at the same amino acid residue, p.(Arg225Pro), was associated with multifocal ectopic Purkinje-related premature contractions (Ter Bekke et al., 2018) and severe cardiac conduction disturbances (Bezzina et al., 2003).

The c.2024-11T > A mutation leads to abolition of the acceptor splice site and creates a cryptic site upstream in SCN5A, and was identified by our team in a patient presenting with dizziness and syncope (Mak et al., 2018). The c.2042A > C missense mutation leads to the amino acid change, H681P, between domains I and II. We have previously reported this case of a fever-induced type 1 Brugada pattern with positive flecainide test but negative EPS (Mok et al., 2003). No syncope or arrhythmic events were observed on follow-up. Nevertheless, functional characterization demonstrated that this mutation led to negative shifts in the steady-state activation and inactivation curves, but had no effect on the recovery from inactivation, which together reduced the sodium current (Mok et al., 2003). The c. 4279G > T mutation was previously reported by us for the first time in association with BrS with recurrent VF (Li et al., 2017). This mutation was previously associated with malignant VT/VF after lidocaine use in acute myocardial infarction (Xiong et al., 2014). The c. 5689C > T mutation in exon 28 leads to the R1897W amino acid change. It was previously linked to early onset lone atrial fibrillation (Olesen et al., 2012) but not a disease-causing mutation in long QT syndrome with minimal effects on the QT interval (Ghouse et al., 2015). This study extends its association to BrS for the first time. The c.429del mutation leads to the Asn144Thrfs^∗^57 frameshift in SCN5A.

Finally, we also identified a novel mutation in CACNA1C in a patient with suspected BrS. The calcium current is mediated by L-type calcium channels (LTCC). Each LTCC consists of four protein subunits α1 (CACNA1C), β2 (CACNB2), α2 (CACNA2D), and δ (CACNA2D). Similar to SCN5A mutations, Antzelevitch et al. suggested that loss-of-function mutations in these genes precipitate abnormal trafficking, reduced expression or function of LTCC, leading to reduced calcium influx current during phase 2 of the cardiac action potential (Antzelevitch et al., 2007; Burashnikov et al., 2010). As a result, BrS secondary to the reduced functionality of LTCCs are associated with shorter QT intervals compared to classical SCN5A mutation BrS where QT interval remains unaltered. The c.5862_5873del mutation was previously classified as likely benign.

## Limitations

Several limitations of this study should be noted. Firstly, this was a retrospective study without standardization of the genetic testing performed. These patients underwent SCN5A testing without next generation sequencing (NGS) of their entire genomes. Therefore, contributions from mutations in other genes such as SCN10A could not be identified. Indeed, a study from Japan of 40 Japanese probands who were clinically suspected with BrS and were negative for mutations in major BrS-related genes were found to have mutations in SCN10A (Fukuyama et al., 2016). One patient in the cohort had CACNA1C and other genes tested only because the son had died suddenly from sudden nocturnal death. Future studies should re-examine these patients using NGS. Finally, given that this was a clinical study, it was not possible to study the effects of the respective genetic mutations on function, expression or membrane trafficking. Future studies should examine ion channel activation, inactivation and recovery properties in patch clamping studies.

## Conclusion

This study identified novel mutations in SCN5A in a Chinese cohort of BrS patients. Future studies are needed to determine their effects on sodium channel function, expression or trafficking, and to test for mutations in other disease-causing genes in BrS.

## Data Availability Statement

The raw data supporting the conclusions of this article will be made available by the authors, without undue reservation.

## Ethics Statement

The studies involving human participants were reviewed and approved by The Joint Chinese University of Hong Kong–New Territories East Cluster Clinical Research Ethics Committee. Written informed consent for participation was not required for this study in accordance with the national legislation and the institutional requirements.

## Author Contributions

GT contributed to the study conception, study design, data analysis, data interpretation, statistical analysis, manuscript drafting, and manuscript revision. SL, TL, HY, IW, CM, and NM contributed to the data analysis, data interpretation, statistical analysis, and manuscript revision. WW contributed to the study conception, study design, study supervision, data analysis, data interpretation, statistical analysis, manuscript drafting, and manuscript revision. All authors contributed to the article and approved the submitted version.

## Conflict of Interest

The authors declare that the research was conducted in the absence of any commercial or financial relationships that could be construed as a potential conflict of interest.

## Footnotes

1
https://cardiodb.org/APPRAISE/

2
http://exac.broadinstitute.org/
